# Association between Timing of Surgical Intervention and Mortality in 15,813 Acute Pancreatitis

**DOI:** 10.1155/2020/1012796

**Published:** 2020-05-16

**Authors:** Lan Lan, Jiawei Luo, Xiaoyan Yang, Dujiang Yang, Mengjiao Li, Fangwei Chen, Nianyin Zeng, Xiaobo Zhou

**Affiliations:** ^1^West China Biomedical Big Data Center, West China Hospital, Sichuan University, Chengdu 610041, China; ^2^Department of Gastrointestinal Surgery, West China Hospital, Sichuan University, Chengdu 610041, China; ^3^West China School of Public Health, Sichuan University, Chengdu 610041, China; ^4^Department of Instrumental and Electrical Engineering, Xiamen University, Fujian 361005, China; ^5^School of Biomedical Informatics, University of Texas Health Science Center at Houston, Houston 77030, USA

## Abstract

**Objective:**

In order to find the quantitative relationship between timing of surgical intervention and risk of death in necrotizing pancreatitis.

**Methods:**

The generalized additive model was applied to quantitate the relationship between surgical time (from the onset of acute pancreatitis to first surgical intervention) and risk of death adjusted for demographic characteristics, infection, organ failure, and important lab indicators extracted from the Electronic Medical Record of West China Hospital of Sichuan University.

**Results:**

We analyzed 1,176 inpatients who had pancreatic drainage, pancreatic debridement, or pancreatectomy experience of 15,813 acute pancreatitis retrospectively. It showed that when surgical time was either modelled alone or adjusted for infection or organ failure, an L-shaped relationship between surgical time and risk of death was presented. When surgical time was within 32.60 days, the risk of death was greater than 50%.

**Conclusion:**

There is an L-shaped relationship between timing of surgical intervention and risk of death in necrotizing pancreatitis.

## 1. Introduction

Indications for surgical intervention of acute pancreatitis (AP) are secondary infections of the pancreas, secondary infections, or compression symptoms, mainly including the pancreas or peripancreatic symptoms or necrosis of secondary infections and organ failure. It is well known that early debridement is associated with higher morbidity and mortality, and recommendations are to delay by at least 4 weeks after the acute pancreatitis episode. Recommendations of guidelines for surgical timing of necrotizing pancreatitis from United States, United Kingdom, Italy, Finland, and Japan are delayed as far as possible, without recommendations for individuals [1–6]. Those recommendations lacking details could result in a large difference in the selection of best surgical timing in practice.

Previous studies [7, 8] on the timing of surgical interventions mostly calculated the time from admission. The time of admission of each patient was susceptible to a variety of factors, such as economic factors and availability of medical resources. Because of the big difference of the time before admission, there is often a certain error based on the time of admission. A more reasonable evaluation should be calculated from the onset of AP (the time of onset of abdominal pain). Additionally, previous studies were mostly qualitative research. A prospective study of 223 patients with well-defined early and late intervention with a subgroup analysis with multiorgan failure and infected necrosis was used [8]. However, they cannot continuously give the risk of death corresponding to a certain point in time. Infection and organ failure have been used as key factors in determining whether or not to undergo surgery and are considered the determinants of mortality for the patients with necrotizing pancreatitis [9, 10]. It was observed that organ failure was more likely to determine mortality in AP [11, 12]. While a prospective cohort study from the Netherlands showed that there were no associations between infection, onset of organ failure, duration of organ failure, and mortality in the patients with necrotizing pancreatitis [13]. What is more, pancreatic amylase is one of the criteria for the diagnosis of AP [14]. High-density lipoprotein within 48 hours after admission is a good predictor of the severity of AP [15], so that the effect of severity can be adjusted by early high-density lipoprotein. White blood cell count on admission is a good indicator of infection, and it can be used to adjust the impact of infection on mortality [16]. Creatinine is the diagnostic criteria for renal failure [14]. Collecting this information prospectively is labor intensive, which often results in a small sample size. Therefore, it is critical that this information can be obtained from Electronic Medical Record (EMR) without extra cost to be researched based on a large sample size.

Therefore, we applied a generalized additive model to quantitate the relationship between surgical time (from the onset of AP to first surgical intervention) and risk of death for 15,813 inpatients diagnosed with AP from EMR, as well as adjusting for demographic characteristics, infection, organ failure, and important lab indicators.

## 2. Materials and Methods

### 2.1. Study Setting and Population

The surgical approach for necrotizing pancreatitis can be classified into three categories: drainage, pancreatectomy, and pancreatic necrotic tissue removal plus extensive drainage [5]. Therefore, we defined study patients as follows: (1) diagnosis with AP on admission based on ICD codes (ICD-9: 577.0, ICD-10: K85) and (2) having at least one surgical intervention experience including pancreatic drainage, pancreatic debridement, or pancreatectomy in a same encounter. At the beginning, 15,813 patients diagnosed with acute pancreatitis were included. After extracting surgical records of the patients, 1,176 patients were included finally (see Figure 1). This study retrospectively collected data of patients with AP and followed the STROBE guidelines [17] for observational studies. The research protocol was approved by the ethics review board of West China Hospital of Sichuan University, and the need for informed consent was waived owing to the retrospective nature of the study.

### 2.2. Data Collection and Definitions

After admission, all patients diagnosed with AP from West China Hospital of Sichuan University initially received traditional treatment. The etiology for patients was main biliary, alcohol abuse, and others. When abdominal pain, severe clinical deterioration, or development of clinical signs of sepsis persisted or recurred, the CECT was performed. Patients with confirmed or suspected infected necrosis were advised to receive surgical intervention based on the CT results. Then, experienced surgeons discussed the case with the radiologist to decide the type and time for surgical intervention, which delayed as much as possible after four weeks from the onset. When patients had persistent clinical manifestations of sepsis, prompt surgical intervention was considered. The data were retrospectively extracted from EMR of West China Hospital of Sichuan University from 2010 to 2018, including demographic characteristics, lab tests, vital signs, and death information. If it was positive for the bacteria in the pancreas or peripancreatic drain, pus, or secretions, the patient was infected. Respiratory failure was defined as the partial pressure of oxygen in blood gas analysis less than 60 mmHg or the use of a ventilator. Circulatory failure was defined as diastolic blood pressure less than 60 mmHg or systolic blood pressure less than 90 mmHg and the use of vasoactive drugs. Kidney failure was defined as creatinine greater than 177 *μ*mol/L. The time from the onset of AP to admission was asked by physicians. The lab test results were extracted from the laboratory information system, and the clinical events (vital signs information, etc.) were extracted from the nursing system.

### 2.3. Statistical Analysis

We used a regular expression [18] to extract the patients who had specific surgical intervention experience and the onset of AP from the clinical notes of EMR in the patients diagnosed with AP on admission. We explored the difference between died and survived inpatients diagnosed with AP after the specific surgical intervention. The baselines of the two groups were compared, including important lab indicators, infection, and organ failure. *t*-test and Chi-square test were used to evaluate the difference between the two groups.

Considering that the relationship between many clinical factors and risk of death are often not linear and the generalized additive model [18] allows each variable to be put in the model in different nonlinear forms, the generalized additive model was used to explore the association between the timing of surgical intervention and risk of death, controlling the potential confounding factors like infection and organ failure. We assumed that the death of the patients obeys the Bernoulli distribution. The formula of the generalized additive model is as follows: *g*(*Y*_*i*_) = *α* + *f*(*x*_1*i*_) + *f*(*x*_2*i*_) + ⋯, where *Y* is death or not, *a* is the intercept, *x* is the independent variable, *i* indicates the *i*th patient, and *f* is the nonlinear function of independent variable. *f* is a smooth cubic spline regression function formulated as *s*(·) in this study. The backfitting method was used to evaluate the model, and the hyperparameter was selected by the Akaike information criterion (AIC). Based on the adjustment of demographic characteristics and important lab indicators, we first adjusted for infection, secondly adjusted for organ failure, and finally modelled surgical time lonely. When a variable with missing values was to be used, the patient with the missing value was deleted. It is statistically significant if the *P* value is less than 0.05. All data analyses were done in the R software.

## 3. Results

### 3.1. Baseline Characteristics

In this study, 1,176 patients with a mean age of 45.57 ± 12.72 years and 780 (66.33%) males who had surgical intervention (pancreatic drainage, pancreatic debridement, or pancreatectomy) in 15, 813 patients diagnosed with AP on admission were analyzed. The number of patients with respiratory failure, circulatory failure, and kidney failure before surgical intervention was 36 (3.06%), 522 (44.39%), and 171 (14.54%), respectively. There were 463 (39.37%) patients infected. The time from the onset of AP to admission and first surgical intervention was 23.05 ± 35.42 days and 34.43 ± 34.95 days, respectively. The total hospital stay was 31.54 ± 25.03 days. Sixty-two (5.27%) patients after surgical intervention died in the hospital.

The baselines between died and survived patients after surgical intervention were compared. There was no difference between the two groups with respect to age and gender. High-density lipoprotein on admission of survived patients was a little higher than that of died patients. Died patients were 2.45 times and 2.44 times than survived patients for amylase on admission and maximum preoperative creatinine, respectively. Their white blood cell count on admission looked similar. The proportion of infection and organ failure in the death group was higher than that in the surviving group except for respiratory failure without statistical difference. The time from the onset of AP to admission and surgical intervention of died patients was shorter than that of survived patients, while total hospital stay was longer without statistical significance (see Table 1).

### 3.2. Modelling Surgical Time and Mortality Adjusted for Infection

Firstly, we modelled surgical time and mortality adjusted for infection, as well as other covariates. The formula is as follows: logit(*Y*_*i*_) = *α* + *s*(*x*_1*i*_, *β*_1_) + *s*(*x*_2*i*_, *β*_2_) + *β*_3_*x*_3*i*_ + *β*_4_*x*_4*i*_ + *s*(*x*_5*i*_, *β*_5_) + *s*(*x*_6*i*_, *β*_6_) + *s*(*x*_7*i*_, *β*_7_), where *x*_1_ is the time from the onset of AP to surgical intervention, *x*_2_ the is age, *x*_3_ is the gender, *x*_4_ is infection or not, *x*_5_ is the high-density lipoprotein on admission, *x*_6_ is the amylase on admission, and *x*_7_ is the white blood cell count on admission (*n* = 708, *R*^2^ = 18.2%). Amylase, high-density lipoprotein on admission, and surgical time had statistical association with death adjusted for age, gender, infection, and white blood cell count on admission (see Table 2).

We further analyzed the independent relationships between risk factors and risk of death.  Figure 2 shows that there was a roughly L-shaped relationship between the time from the onset of AP to surgical intervention and risk of death, which indicates that premature surgery has a higher risk of death than postponed surgery. The older, the smaller the high-density lipoprotein or the higher the amylase on admission and the higher the risk of death. The risk of death in white blood cell count on admission was first rising and then falling. The shaded area represents the 95% confidence interval.

### 3.3. Modelling Surgical Time and Mortality Adjusted for Infection and Organ Failure

Secondly, we modelled surgical time and mortality adjusted for infection and organ failure, as well as other covariates. The formula is as follows: logit(*Y*_*i*_) = *α* + *s*(*x*_1*i*_, *β*_1_) + *s*(*x*_2*i*_, *β*_2_) + *β*_3_*x*_3*i*_ + *β*_4_*x*_4*i*_ + *s*(*x*_5*i*_, *β*_5_) + *s*(*x*_6*i*_, *β*_6_) + *s*(*x*_7*i*_, *β*_7_) + *s*(*x*_8*i*_, *β*_8_) + *β*_9_*x*_9*i*_ + *β*_10_*x*_10*i*_ + *β*_11_*x*_11*i*_, where *x*_1_ is the time from the onset of AP to surgical intervention, *x*_2_ is the age, *x*_3_ is the gender, *x*_4_ is infection or not, *x*_5_ is the high-density lipoprotein on admission, *x*_6_ is the amylase on admission, *x*_7_ is the white blood cell count on admission, *x*_8_ is the maximum preoperative creatinine, *x*_9_ is respiratory failure or not, *x*_10_ is circulatory failure or not, and *x*_11_ is kidney failure or not (*n* = 708, *R*^2^ = 31.5%). Amylase on admission had a statistical association with death adjusted for surgical time, age, gender, infection, organ failure, and other lab indicators (see Table 3).

The independent relationships between risk factors and risk of death were also analyzed.  Figure 3 shows that after the inclusion of more variables, the relationship between surgical time, age, high-density lipoprotein, amylase, and white blood cell count and risk of death remained similar. The risk of death was high in a specific range and low in both ends of creatinine.

### 3.4. Modelling Surgical Time and Mortality

Finally, we developed a model adjusted for age, gender, and high-density lipoprotein formulated as logit(*Y*_*i*_) = *α* + *s*(*x*_1*i*_, *β*_1_) + *s*(*x*_2*i*_, *β*_2_) + *β*_3_*x*_3*i*_ + *s*(*x*_4*i*_, *β*_4_), where *x*_1_ is the time from the onset of AP to surgical intervention, *x*_2_ is the age, *x*_3_ is the gender, and *x*_4_ is the high-density lipoprotein on admission, to find the relationship between surgical time and risk of death. Age and gender, as well as high-density lipoprotein, were used to adjust for basic characteristics and severity of AP, respectively. Based on the premise, the relationship between surgical time and risk of death in the infected and noninfected groups was also studied. In this section, we applied generalized additive model based on different samples: all patients (*n* = 1, 144, *R*^2^ = 7.92%), infected patients (*n* = 463, *R*^2^ = 5.96%), and noninfected patients (*n* = 681, *R*^2^ = 13.40%). There was a statistical correlation between surgical time and mortality in the three groups.

Figure 4 shows that the relationship between surgical time and death was similar among all, infected, and noninfected patients. Because the risk of death was very low after 100 days of surgical time, we only figured out the surgical time within 100 days. The relationship between surgical time and death was the same in the infected and noninfected patient groups. Surgical time 32.60, 32.84, and 36.55 days in all, infected, and noninfected patients, respectively, had 50% risk of death. The risk of death would be more than 50% if the surgical time was less than the thresholds.

## 4. Discussion

This study investigated the relationship between surgical timing and death in necrotizing pancreatitis based on a large sample of EMR. The inpatients of AP with the specific surgery (pancreatic drainage, pancreatic debridement, or pancreatectomy) were modelled, who were almost patients with necrotizing pancreatitis. According to our best knowledge, there is no quantitative study between the timing of surgical intervention (from the onset of AP to first surgical intervention) and risk of death in necrotizing pancreatitis. This study is the first case. There is an L-shaped relationship between surgical time and risk of death in necrotizing pancreatitis, showing that premature surgery carries a higher risk of death among patients with necrotizing pancreatitis. This kind of relationship is still robust after sensitivity analyses.

In descriptive analyses, the time from the onset of AP to surgical intervention, time from the onset of AP to admission, high-density lipoprotein on admission, amylase on admission, maximum preoperative creatinine, infection, circulatory failure, and kidney failure had a statistical difference with respect to death. These variables were further put in the model at the same time to check if there was a real impact on death. In the first model incorporating infection and other covariates, results showed that the lower high-density lipoprotein on admission, the higher the risk of death, which is consistent with previous study [15]. And for the second model inclusion of infection and organ failure as well as other covariates, the relationship between the two was similar, but it was not statistically significant. Amylase was statistically significant in the inclusion of infection or organ failure. The higher the amylase, the higher the risk of death, and risk of death exceeded 50% when amylase was over 175.54 mmol/L. The risk of death for white blood cell count was first rising slowly and then decreasing quickly. One of the most possible reasons is that the doctor will give an antibiotic treatment to control the white blood cell count in a normal range and reduce the probability of infection when the white blood cell count exceeds 10 × 10^9^/L. Therefore, the risk of death would decline when the white blood cell count exceeds 10 × 10^9^/L. In both models, infection was not statistically significant, which has similar results with Guo et al. [11] Our proposed model can deal with a collinear independent variable. Respiratory failure, circulatory failure, kidney failure, and creatinine were not statistically significant after including in the second model, consistent with the findings of the Dutch Pancreatitis Study Group [13]. However, we found that risk of death was low when creatinine was too low or too high, and risk of death was higher than 50% with creatinine ranging from 73.55 to 818.06 *μ*mol/L. For the relationship between age and death, although there was no statistical difference in the first and second models, it presented increased risk of death with increase in age.

Some covariates may not have statistical differences, but as can be seen from previous figures, these variables have a regularity with risk of death, and our model gave a threshold of 50% risk of death, which is worthy of attention of surgeons. After adjusting for infection, of surgical time and death that was still statistically significant. But after adjusting for organ failure, there was no statistical significance. No statistical difference does not mean that there is no real association between the two. Statistical difference is related to many factors such as the choice of independent variables and sample size. Therefore, in order to find out the relationship between surgical time and risk of death, we finally modelled surgical time adjusted for age, gender and high-density lipoprotein on admission since demographic factors can also be utilized as predictors of inpatients mortality in AP [19]. It was found that when surgical time was either modelled alone or adjusted for infection or organ failure, an L-shaped relationship was presented. Surgical time was within 32.60 days, the risk of death was greater than 50%. Not only that, but this study also obtained the mortality risk corresponding to the timing of surgical intervention at each time point. Although the relationship between surgical time and death was similar in the infected and noninfected groups, surgical time of the infected group (32.84 days) was earlier than that of the noninfected group (36.55 days) at 50% risk of death, and risk of death from early surgery for the noninfected group was 77%, which was a little higher than that (72%) of the infected group.

Although amylase is one of the criteria for the diagnosis of acute pancreatitis, the relationship between amylase and the severity of acute pancreatitis is rarely reported. However, there are many reasons for the patients who have abnormal levels of amylase in their blood, including sudden inflammation of the pancreas, long-term inflammation of the pancreas, fluid-filled sac around the pancreas, pancreatic cancer, inflammation of the gallbladder, and kidney problems. The results of this study showed that the higher the amylase, the higher the risk of death. The reason for this result may be that there are other diseases that also cause high amylase, except acute pancreatitis. Under the combined effect of various diseases, the risk of death is increased. If considering the effects separately, the quantitative relationships between different surgical time and other covariates at different levels and risk of death can be a good reference for surgeons. The results of this work are based on EMR. Other hospitals can use this research strategy to obtain preliminary results and then conduct prospective design. Therefore, this study provides an important prerequisite for a prospective study.

However, there are still some limitations in this study. The data is retrospectively extracted from EMR, and the performance of the model is strongly correlated with the quality of the data. The death cases were recorded during hospitalizations, and the cause of death was not available based on EMR. Due to the Chinese cultural characteristics, some patients who do not want to die in the hospital will be discharged early and those deaths will not be recorded in the EMR. Therefore, in this study, mortality was underestimated, and its relationship with surgical time was also underestimated. On the other hand, since the generalized additive model cannot analyze the interaction between variables, there may be interactions between variables. It is the limitation of the model itself.

## 5. Conclusions

In conclusion, by applying the generalized additive model, we obtained the relationship between surgical time (from the onset of AP to first surgical intervention) and risk of death in the case of controlling demographic characteristics, infection, organ failure, and important lab indicators in necrotizing pancreatitis. There is an L-shaped relationship between timing of surgical intervention and risk of death in necrotizing pancreatitis, providing an important reference for surgeons when making surgical decisions.

## Figures and Tables

**Figure 1:** Flow diagram of this study.

**Figure 2:** The relationship between risk of death and five risk factors.

**Figure 3:** The relationship between risk of death and six risk factors.

**Figure 4:** The relationship between risk of death and surgical time ((a1) is for all patients, (a2) is for infected patients, and (a3) is for noninfected patients).

**Table 1:** Baselines between died and survived patients after surgical intervention.

Characteristics	Died (*n* = 62)	Survived (*n* = 1,114)	*P*
Age (year, mean (SD))	48.21 (13.32)	45.43 (12.67)	0.094
Male, *n* (%)	39 (62.90)	741 (66.52)	0.654
Lab indicator			
High-density lipoprotein on admissionª (mmol/L, mean (SD))	0.43 (0.31)	0.60 (0.37)	0.001^∗^
Amylase on admissionª (U/L, mean (SD))	635.79 (647.36)	259.47 (537.16)	<0.001^∗^
White blood cell count on admissionª (10^9^/L, mean (SD))	11.92 (5.25)	10.82 (6.51)	0.208
Maximum preoperative creatinineª (*μ*mol/L, mean (SD))	217.34 (190.20)	89.10 (103.13)	<0.001^∗^
Infection, *n* (%)	37 (59.68)	426 (38.24)	0.001^∗^
Organ failure before surgical intervention			
Respiratory failure, *n* (%)	2 (3.23)	34 (3.05)	1.000
Circulatory failure, *n* (%)	49 (79.03)	473 (42.46)	<0.001^∗^
Kidney failure, *n* (%)	37 (59.68)	134 (12.03)	<0.001^∗^
Time from the onset to admission (day, mean (SD))	11.55 (14.96)	23.69 (36.12)	0.009^∗^
Time from the onset to surgical intervention (day, mean (SD))	23.03 (16.33)	35.07 (35.60)	0.008^∗^
Total hospital stay (day, mean (SD))	32.21 (27.54)	31.50 (24.90)	0.829

SD: standard deviation; *n* (%): number and percentage; ^∗^ indicates statistical significance; ^a^Different missing rates 2.7%, 8.3%, 4.2%, and 2.7% for high-density lipoprotein, amylase, white blood cell count on admission, and maximum preoperative creatinine, respectively.

**Table 2:** Model results between surgical time and mortality adjusted for infection.

Covariates	*β*	SD	*Z* or *χ*^2^	*P*
Intercept	-4.117	0.502	-8.200	<0.001^∗^
*s* (time from the onset to surgical intervention)	-	-	4.282	0.042^∗^
*s* (age)	-	-	0.836	0.563
Male	-0.300	0.453	-0.662	0.508
Infection	0.597	0.456	1.308	0.191
*s* (high-density lipoprotein)	—	—	7.037	0.022^∗^
*s*(amylase)	-	-	20.197	<0.001^∗^
*s* (white blood cell count)	-	-	0.952	0.575

‘-' no traditional slope concept in this study; ^∗^ indicates statistical significance.

**Table 3:** Model results between surgical time and mortality adjusted for infection and organ failure.

Covariates	*β*	SD	*Z* or *χ*^2^	*P*
Intercept	-4.586	0.608	-7.541	<0.001^∗^
*s* (time from the onset to surgical intervention)	-	-	1.489	0.235
*s* (age)	-	-	0.919	0.459
Male	-0.895	0.516	-1.734	0.083
Infection	0.531	0.505	1.051	0.293
*s* (high-density lipoprotein)	-	-	1.739	0.268
*s* (amylase)	-	-	12.749	0.005^∗^
*s* (white blood cell count)	-	-	0.697	0.665
*s* (creatinine)	-	-	2.845	0.408
Respiratory failure	-1.794	1.409	-1.273	0.203
Circulatory failure	0.858	0.498	1.722	0.085
Kidney failure	1.306	0.760	1.718	0.086

‘-' no traditional slope concept in this study; ^∗^ indicates statistical significance.

## Data Availability

The datasets generated during and/or analyzed during the current study are available from the corresponding author on reasonable request.
